# Toxicological and Teratogenic Effect of Various Food Additives: An Updated Review

**DOI:** 10.1155/2022/6829409

**Published:** 2022-06-24

**Authors:** Saseendran Sambu, Urmila Hemaram, Rajadurai Murugan, Ahmed A. Alsofi

**Affiliations:** ^1^Department of Food Technology, Faculty of Life and Allied Health Sciences, Ramaiah University of Applied Sciences, Bengaluru, Karnataka, India; ^2^Department of Pharmacy, Faculty of Medical Sciences, Aljanad University for Science and Technology, Taiz, Yemen

## Abstract

Scientific evidence is mounting that synthetic chemicals used as food additives may have harmful impacts on health. Food additives are chemicals that are added to food to keep it from spoiling, as well as to improve its colour and taste. Some are linked to negative health impacts, while others are healthy and can be ingested with little danger. According to several studies, health issues such as asthma, attention deficit hyperactivity disorder (ADHD), heart difficulties, cancer, obesity, and others are caused by harmful additives and preservatives. Some food additives may interfere with hormones and influences growth and development. It is one of the reasons why so many children are overweight. Children are more likely than adults to be exposed to these types of dietary intakes. Several food additives are used by women during pregnancy and breast feeding that are not fully safe. We must take specific precaution to avoid consuming dangerous compounds before they begin to wreak havoc on our health. This study is intended to understand how the preservatives induce different health problem in the body once it is consumed. This review focuses on some specific food additives such as sodium benzoate, aspartame, tartrazine, carrageenan, and potassium benzoate, as well as vitamin A. Long-term use of food treated with the above-mentioned food preservatives resulted in teratogenicity and other allergens, according to the study. Other health issues can be avoided in the future by using natural food additives derived from plants and other natural sources.

## 1. Introduction

Food additives are used in the product and processing of nearly all types of food to give desirable rates. Simply said, it is a material that is added to food to ameliorate its flavor, appearance, or other desirable characteristics. Some of the food additives are listed in Table 1. Food additives are defined by the US Public Exploration Council's food protection commission as “a substance or a mixture of substances that is present in a food as a result of an aspect of product, processing, storage, or packaging.” Teratogens are chemicals that, when exposed to a pregnant woman, can cause physical or functional defects in a human embryo or fetus. Its examples include alcohol and cocaine. The length of exposure, the amount of teratogenic material present, and the stage of development of the embryo at the moment of exposure all have an effect on the embryo [1].

Teratogens can affect an embryo in a variety of ways, including physical deformities and behavioural or mental disorders and a reduction in the child's intellectual quotient. It can also lead to problems including unseasonable labor, robotic revocations, and deliveries and detriment embryo. Physical agents, metabolic circumstances, infection, and incipiently drugs and chemicals are the four orders of teratogens [2].

Food complements are composites that food manufacturers add to food in small quantities during product or processing to ameliorate the food's organoleptic parcels similar as flavor, appearance, and taste [3]. They contribute to the food's shelf life by icing product thickness, healthiness, and newness. They make a variety of accessible foods available without the stress of grocery shopping or cuisine on a diurnal base. The complements must be added in precise quantities and should be within the diurnal consumption limits.

Some complements, similar as those used to save food, have been used for glories pickling (preservation with ginger) and salting, the preservation of sweets, and the usage of sulphur dioxide in wines. With the preface of reused foods in the alternate half of the twentieth century, numerous further complements were introduced in the alternate part of the twentieth century. Both natural and artificial origins have been added [4].

Food complements can be employed in a number of ways, both directly and laterally. Direct complements are those that are added to foods for a definite purpose, whereas circular complements are those that are added after the fact during manufacturing, puddings, yoghurt, and biting goods [5].

Numerous food complements are listed on the component marker of a product. Some food complements may enter the food in trace quantities during quilting, storehouse, or handling that are known as circular food complements. Some colourings, similar as erythrosine, are exemplifications (red); Colourants like erythrosine (red) and canthaxanthine (unheroic orange) give dishes a nice appearance that attracts guests despite the fact that they do not provide any nutrients [6]. Some food complements that show teratogenicity are described below.

## 2. Methodology

Required data were searched/collected from the online databases as described by researcher [7] including Wiley, Google, PubMed, Google Scholar, ScienceDirect, and Scopus. Keywords used in search are in toxicological evaluations, food additives, and teratogenicity. Latest published data were selected.

## 3. Results and Discussion

### 3.1. Preservatives as Teratogens

A preservative is any material able to prevent, slow down, or stop the growth of microorganisms, as well as any food deterioration caused by microorganisms. Preservatives can be antimicrobial, inhibiting the growth of bacteria or fungi, or antioxidants, which operate similarly to oxygen absorbers by inhibiting the oxidation of food constituents. Traditional preservatives also include natural compounds such as sugar, ginger, alcohol, and diatomaceous earth. Calcium propionate, sodium nitrate, sodium benzoate, sodium nitrite, sulfites (sulphur dioxide, sodium bisulfite, potassium hydrogen sulfite, etc.), and disodium are examples of common chemical preservatives [8]. The preservatives that cause teratogenicity are noted below.

#### 3.1.1. Sodium Benzoate

Sodium benzoate (Figure 1) is a synthetic food preservative, which is extensively used in food, medicinal, and cosmetics diligence. The chemical is a sodium salt of benzoic acid that is safe to eat and apply to the skin. It should not be used in some acidic products because it can interact with other chemicals to induce dangerous composites, but it is not poisonous or irritable to tissue. It dissolves easily in water, and its inclusion in food is approved as it is able to prevent the growth of molds and other microbes. The negative effects of sodium benzoate on health have been established, including cellular damage. Numerous research has been conducted in recent years on the use of natural elements with various purposes in food, with some success, but there is still a need to study in the food sector. The teratogenic impact of sodium benzoate is discussed below with the assistance of a study of fetal deformations due to long-term consumption of sodium benzoate in pregnant BALB/c mice [9].

*(1) Mechanism of Action*. A high dosage of sodium benzoate can induce histamine to be released from the body. H1 receptors are affected by mast cell granules and histamine accessible in endothelial cells, leading to a rise in artery diameter leaking of elements of blood plasma and its permeability in the tissues. As a result, it is suitable to assign hemorrhages, and physical tissue damage reported in sodium benzoate affects the skin of embryos by this way. Sodium benzoate enters into blood vessels and interfere with genes, which is invloeved in the synthesis of blood clotting factors [10]. The studies have also shown the cytogenetic goods of benzoic acid sodium salts in lymphocytes [11]. In mice, exposure to methylnitrosourea (MNU) caused proliferating cell damage via macromolecule alkylation and the production of reactive oxygen species (ROS). Elevated ROS levels in mice lowered the severity of retinal abnormalities and, though unknown mechanisms, inhibited fetal Pax-3 gene expression, which is crucial in neural tube development blockage [12]. In proliferating embryonic tissues of rats, increased ROS suppresses the expression of the bcl-2 (antiapoptotic) gene. Rajadurai and Prince (2006) have reported that elevated production of ROS in the biological system showed adverse effects on nuclei acids [13].

Some benzoate derivations, such as SB, appear to be free radical scavengers in humans [14], whereas other mechanisms possibly causing embryonic hemorrhage and eye tissue disorders after PB exposure may result from the induction of potentially harmful ROS situations in embryonic tissues (such as the eye) and inhibit embryonic gene expression, such as Pax-3 or alternative genes required for blood clotting. Our study's findings are related to hyperkalemia, which has been associated to intraventricular hemorrhage in premature neonates. Researchers hypothesized that low systemic blood flow, as measured by lower urine output and K+ secretion, could contribute to the development of hyperkalemia in premature neonates [15]. It is also believed that the hemolytic activity of the limited intraventricular blood clot contributes to an intraventricular K^+^ load surplus [16].

*(2) Adverse Effects*. The current study's findings on the teratogenic effects of sodium benzoate on embryo revealed a variety of defects, including craniofacial deformities. Mandibular hypoplasia and other forms of mandibular hypoplasia are the most common calvarias deformity and vertebral column deformation. Scoliosis and neural tube defects (NTDs) are two examples of this. It had been argued in a study that administering high doses of antibiotics on a daily basis sodium benzoate has the potential to be genotoxic and teratogenic modifications in the neurological system [17]. The other severe impacts also include on growth factors, cell cycle, and gene expression, as well as the fact that it can cause deformations during birth. Food additives in general must be reevaluated as needed in light of new information shifting usage situations and fresh scientific findings information.

#### 3.1.2. Potassium Benzoate

Potassium benzoate (Figure 2) is an odorless white powder made by heating benzoic acid and potassium salt together. Benzoic acid is a naturally occurring chemical found in plants, animals, and fermented foods. It was once made from the benzoin resin of particular tree species, but it is now largely made in factories. Salt beds or minerals are the most common sources of potassium salts. PB is used as a preservative because it prevents bacteria, yeast, and mold from growing. As a result, it is frequently used to increase the shelf life of food, beauty, and skin care goods. The teratogenicity of potassium benzoate is defined by an experiment “Teratogenic Effects of Long-term Consumption of Potassium Benzoate on Eye Development in BALB/c Fetal Mice” [18].

*(1) Mechanism of Action*. It has also been observed that potassium benzoate suppresses intracellular protein and DNA synthesis at doses below 100 pg/ml and over 500 pg/ml. The study found that benzoic acid (200 and 500 pg/ml) increases chromosomal abnormalities, sister chromatid exchanges, and micronucleus prevalence in human cells without changing the medium pH [19]. There is some suggestion that a mutation in the homeobox gene, OTX2, may also be implicated in the development of these symptoms. The expression pattern of the OTX2 gene in human embryo is also linked to bilateral anophthalmia to certain retinal consequences and pigmentary retinopathy [20]. Because PB can be mutagenic, various studies have been done to precisely investigate the potential teratogenic effects of the food preservative, PB, on the embryonic eye development in pregnant mice. The findings showed that pregnant mice exposed to PB experienced severe bleeding of the embryonic eye, a malformed lens, and retinal folds with underdeveloped layers. Because of the complexity of eye development, many congenital anomalies occur, but most of them are not common [21].

Congenital eye abnormalities can be caused by a variety of environmental teratogens. Some studies have found a link between the use of some antiepileptic medicines during pregnancy and congenital eye malformations such as anophthalmia, microphthalmia, or coloboma of the iris or optic disc [22]. Defects in the PAX6 gene expression cause aniridia-like iris abnormalities [23], corneal opacities, and lens-corneal adhesions similar to Peters' anomaly [24]. Detailed histologic examinations of neonatal mice with Peters-like abnormalities indicated that the lens commonly fails to detach from the cornea [25]. Furthermore, the study found that OTX2 loss-of-function mutations are linked to a wide range of ocular phenotypes, from bilateral anophthalmia to mild microphthalmia with retinal abnormalities [26].

Alqahtani et al. have investigated the cytogenetic effects of potassium salts of 1-p-(3-methyltriazeno) benzoic acid in human lymphocytes [7]. There was also a dose-dependent increase in chromosome breakage in human cells after exposure to 1-p-(3-methyltriazeno) benzoic acid potassium salts [27]. Dose-dependent administration of toxicant showed increased toxicity and reaches the saturation level at certain doses. As a result, PB and reduced cell proliferation, as well as PAX6 and OTX2 mutation, delayed normal eye development.

*(2) Adverse Effect*. The potential teratogenic effects of PB on embryonic eye development were investigated in the study. As a result of the exposure of pregnant mice to PB, severe bleeding of the embryonic eye, malformed lenses, and retinal folds with underdeveloped layers were observed. Many congenital defects occur as a result of the intricacy of eye development; however, the majority of them are uncommon [28]. Congenital eye abnormalities can be caused by a variety of environmental teratogens. Some researchers have discovered clear evidence of a link between antiepileptic drug use during pregnancy and congenital eye malformations including anophthalmia and microphthalmia [29].

Mice treated to methyl nitrosourea (MNU) during pregnancy suffered harm to proliferating cells due to macromolecule alkylation and reactive oxygen generation. Increased ROS in mice reduced the severity of retinal problems and blocked fetal Pax-3 gene expression, which is important for neural tube development, through unknown processes [30]. Other mechanisms that may cause embryonic bleeding and eye tissue abnormalities after PB exposure include the generation of potentially harmful ROS levels in embryonic tissues (such as the eye) and the inhibition of embryonic gene expression such as Pax-3 or alternative blood clotting genes. The above findings are comparable to those of hyperkalemia, which has been linked to intraventricular hemorrhage in premature babies. In our research, we discovered that PB-exposed mouse fetuses have significantly reduced weight and crown-rump lengths. Adult mice subjected to 280 and 560 mg/kg/day of PB for 20 days showed no adverse effects. As a result, it is thought that mouse embryos are more vulnerable to PB than adults. The above findings imply that PB has teratogenic effects on mouse fetuses' ocular development. Thus, further detailed investigations on its specific and general impacts are required [31].

### 3.2. Sweeteners as Teratogens

Sweeteners are defined as food additives that are used or intended to be used either to conduct a sweet taste to food or as a tabletop sweetener. They are substances of low energy value that give sweet taste but do not have the calories of carbohydrates or their cariogenic or glycemic goods. Sweeteners are classified as either high intensity or bulk. High-intensity sweeteners retain a sweet taste but are noncaloric, give basically no bulk to food, have lesser agreeableness than sugar, and are thus used at veritably low situations [32].

On the other hand, bulk sweeteners are generally carbohydrates, furnishing energy (calories) and bulk to food. Other sweeteners are used to keep the food's energy (calories) low, and they are typically suggested for diabetic's people, dental decay, and diarrhoea so that the blood sugar situations will not rise. Sweeteners are classified as natural and synthetic. The natural ones are the most nutritional salutary sweeteners like sucrose, fructose, lactose, and maltose. The synthetic sweeteners because of their violent agreeableness are called high energy sweeteners (HPS), e.g., certain proteins and terpenes glycosides like saccharin, cyclamates, aspartame, and acesulfame-K [33].

Artificial sweeteners are substantially man-made chemicals that are not found in nature. Such chemicals can be dangerous to human body. It can cause ingestion and other health-related issues. The most contraversial artificicial sweetner, aspartame (Figure 3) discussed below, may cause neurological damage especially in younder children where brain is still developing. It breaks down in the body to phenylalanine, and it may also contribute to obesity. Its metabolites can be toxic to many organs, although there have been a few investigations on the use of aspartame during pregnancy, which may result in deformities. Using chick embryos as a model, this study investigated how aspartame serves as a teratogenic agent on development. It is noncaloric (4 kcal/g) and not suited for diabetics. Aspartame is also teratogenic and is used as an addition in baking items. The research Teratogenic effect of Aspartame Exposure on Chick Embryonic Development possibly describes the teratogenic effect of aspartame [34].

#### 3.2.1. Mechanism of Action

Despite the Food and Drug Administration's approval of L-aspartyl-L-phenylalanine methyl ester (aspartame), there are still worries about the safety of this commonly used low-calorie sweetener. One source of worry is the potential impact of aspartame on embryo and child development. Because the placenta can concentrate amino acids in fetal plasma, almost twice the concentration seen in the mother's plasma, developing fetuses may be especially vulnerable to the effects of aspartame [35]. Aspartame is rapidly degraded after ingestion into its two main amino acids, phenylalanine (about half of aspartame by weight) and aspartate (about forty percent). Because children have relatively lower body weights, their dose levels in terms of body weight could be significantly higher than adults ingesting equivalent amounts of aspartame-containing meals [36]. Children and infants may be more sensitive to the effects of aspartame than adults due to variations in their physiological responses to its constituent amino acids. Protein synthesis has been demonstrated to be reduced by high amounts of phenylalanine.

During infancy, when brain protein synthesis is critical, the phenylalanine component of aspartame's potential harmful effects may be amplified. When given intraperitoneally at 1000 mg/kg body weight, phenylalanine was demonstrated to reduce protein synthesis in the brains of baby rats [37]. Intraperitoneal injection of phenylalanine (2000 mg/kg body weight) affects protein synthesis in newborn mice, but not in older mice [38]. The reduction in brain protein synthesis has also been linked to high amounts of other amino acids. During brain development, hyperphenylalaninemia can diminish myelin production, as seen by decreased incorporation of methionine into myelin proteins [39], decreased total lipid content, decreased myelin yield, [40], and overall lower brain weight [41]. Aspartame and its constituent amino acids have been studied for their impact on baby development. Infant mice were demonstrated to have brain damage after being intragastrically intubated with high doses of aspartate [42].

The women are deficient in an enzyme that permits them to digest the amino acid phenylalanine, which is a component of aspartame. If they consume aspartame, they may develop excessive levels of phenylalanine in their blood, which can result in birth abnormalities. The cytotoxicity of aspartame-derived methanol and its metabolite formaldehyde adducts was exerted through functional change of proteins and DNA mutations, resulting in brain damage, growth retardation, abnormalities, and death of cells. Further, oxidative stress may be the cause of nuclear damage [43].

#### 3.2.2. Adverse Effect

The total amount of chick embryos in all experimental groups exhibited retardation of brain formation in all three sections, as well as brain flexure (only cephalic flexure and microphthalmia and no branchial flexure), anencephaly, anophthalmia, aberrant cardiac looping, tail degeneration, and node degeneration. Limb buds and somites slow down only half of the body's development [44]. At high aspartame concentrations, there were obvious adverse effects such as growth retardation, shrinkage, tail deformities in developing embryos, and physiological changes [45]. The administration of aspartame to rats implies that aspartame administration during pregnancy slows fetal growth due to cell damage during this time [46]. The outcomes of this study clearly demonstrated that aspartame concentrations increase, resulting in many observable defects and deformities in chick embryonic development at high concentrations. As a result, pregnant women should avoid consuming aspartame for the sake of their own safety.

### 3.3. Stabilizers as Teratogens

These substances help to improve and stabilize food texture, help crystallization (sugar and ice), and keep emulsions and foams stable to make icings on baked goods less sticky, and flavors are encapsulated. Polysaccharides, similar as Arabic gum, are thickeners. Thickeners include polysaccharides such as Arabic gum, agar-agar, alginic acid, starch and its derivatives, carrageenan, and pectin. One noncarbohydrate material that is constantly employed for this purpose is gelatin. Hydrophilic stabilizers and thickeners are diffused in water colloids as a solution [47]. These thicken meals by swelling in hot or cold water. Gravies, pie fillings, cutlet condiments, jellies, puddings, and salad dressings are just the many examples of what you can make. Thickeners are added to make the mix thicker density without affecting its other characteristics significantly. In milk and dairy products, the food additives that cause teratogenicity are discussed below. The stabilizers used in dairy product cause teratogenicity. Carrageenan is one of the examples for stabilizers used in dairy products and its teratogenic effect is noted below.

#### 3.3.1. Carrageenan

Carrageenan (Figure 4) is a type of natural linear sulfated polysaccharide found in red edible seaweeds. Chondrus crispus (Irish moss) is a dark red parsley-like plant that grows adhering to the rocks and is still most important red seaweed utilized for creating the hydrophilic colloids necessary to make carrageenan. Because of their gelling, thickening, and stabilizing qualities, carrageenan is frequently employed in the food business. Because of their high binding to dietary proteins, they are mostly used in dairy and meat products. Carrageenan which mimics the native glycosaminoglycans (GAG) has emerged as a viable candidate in tissue engineering and regenerative medicine applications in recent years [48]. Tissue engineering, wound covering, and medication delivery are the most common applications. Carrageenan is a biopolymer derived from algae that is widely utilized in the food industry to generate gels and emulsions in order to stabilize fat in milk, ice cream, and milkshakes.

*(1) Mechanism of Action*. In the current study's experimental conditions, lambda carrageenan has a teratogenic effect on chicken embryos. These findings are consistent with those of Hunt (‘51), who discovered that injecting sucrose into albumen caused a variety of abnormalities of the hen's egg. Some sugars (mono-, di-, and trisaccharides) can cause abnormalities in chicken embryo. Carrageenan induced defects in chick embryos that were similar to those induced by a number of other teratogenic substances. The current findings reinforce the notion that the neural tube and embryonic axis are extremely vulnerable to teratogenic chemicals, while it is still in the early phases of development [49]. Furthermore, because lambda carrageenan elicited anomalies that were comparable to or identical to those provoked by a variety of other chemical and physical agents, it can be assumed that suggested that the pathophysiology of most, if not all, of them is governed by a similar mechanism.

The teratogenic impact of lambda carrageenan on the chick embryo can be explained by at least two mechanisms: (1) carrageenan can bind to cell surfaces, preventing regular cell activity and morphogenesis; or (2) this polygalactoside could be broken down into simple sugars like galactose, which has teratogenic properties. Both hypotheses are supported by evidence. In terms of carrageenan's direct influence on cell surfaces, cell-surface components play a role in cell-to-cell contacts and embryonic morphogenesis.

In terms of carrageenan's direct influence on cell surfaces, cell-surface components are involved in cell-to-cell contacts and embryonic morphogenesis [50]. On the other hand, erythrocytes have been shown to bind sulfated polysaccharides like carrageenan [51]. There is evidence that surface glycosyltransferases catalyse the glycosylation of the terminal end of the matching sugar chain [52]. Carrageenan may interfere with the linking of the terminal sugars of glycoconjugates on the cell surface.

*(2) Adverse Effects*. Strong acid phosphatase activity has been related to a process mediated by carrageenan degradation products in the chick's blastoderm border, with distinct enzymatic activity in yolk globules, implying that the latter corresponds to specific structures [53]. Galactose was likely released as a result of the breakdown of carrageenan in the embryo or in cells of the area vacuoles, or both, causing the abnormalities reported therein. The lambda carrageenan-injected group had partial duplication of the body, aberrant trunk flexures, anencephaly, a severely deformed brain, thickening of the neural tube wall, and an irregular neural tube lumen with segmentary occlusion [54]. Carrageenan caused abnormalities in chick embryos that were similar to those caused by a variety of other teratogenic chemicals. The current findings back up the theory that the neural tube and embryonic axis are extremely vulnerable to teratogenic chemicals at early stages of development [55].

### 3.4. Colouring Agents as Teratogens

Colour additives are any dye, pigment, or material that can be used to colour food and cosmetics (either alone or in combination with other substances) [56]. Colourants are compounds added to colour food or correct the colour of food, according to the Codex Alimentarius Commission (CAC). Furthermore, colourants are used to restore the natural colour of the food that has been lost during processing and storage, to improve the current colour, to strengthen the weak colour, to colour food that is truly colourless, and to win customers by concealing substandard quality [57]. Natural and synthetic sources are used to categorise them. Plant and animal animals, as well as microbes, produce natural colouring substances, for example annatto, anthocyanin, carotenes, and lycopenes. Synthetic colourants are compounds that are not found in nature and are created through chemical synthesis: Allura red, tartrazine, erythrosine, sunset yellow, and more colours [58].

Synthetic food colourants outperform natural food colourants in terms of colouring ability, colour tone, colour distribution, brightness, stability, and ease of use [59]. Synthetic food colourants, on the other hand, have long been thought to have a negative impact on human health and children's behaviour, such as behavioural disorders, hyperactivity, and attention impairments, all of which exhibit significant individual differences in children [60]. The teratogenic effect of tartrazine is discussed below.

#### 3.4.1. Tartrazine

Tartrazine (Figure 5) is a chemical dye having the formula 3-carboxy-5-hydroxy-1(p-sulfophenyl)-4-carboxy-5-hydroxy-1(p-sulfophenyl)-4-carboxy-5-hydroxy-1(p-sulfophenyl)-4-carboxy-5-hydroxy-1(p-sulfophenyl)-4-carboxy-5-hydroxy-1(p-sulfophenyl)-4-carboxy-5- hydroxy-1(p-sulfophenyl)-4-carboxy-5-hydroxy-1((sulfophenylazo) pyrazolone E 102, FD & C Yellow No. 5 [61]. To produce a yellow colour, it is commonly used as a food colourant in sweets, juices, jams, mustard, and sodas [62]. The work “Embryotoxic and Teratogenic Effects of Tartrazine in Rats” describes tartrazine's teratogenicity [63].

*(1) Mechanism of Action*. TAZ is the most commonly used food dye. TAZ causes hepatonephrotoxicity and changes many metabolic characteristics in experimental animals at doses several times greater than its ADI for humans, according to past studies [64]. Furthermore, TAZ causes leucocyte DNA damage in rat liver and kidneys, as well as severe cellular changes, which could have negative health consequences [65]. The stage of embryonic development is crucial in defining the embryo's susceptibility to the drug and, as a result, its response pattern.

A recent study found that nearly all medicines given during pregnancy enter the fetal blood via passive diffusion to some extent [66]. Lipid solubility and molecule size are the two most important elements that influence placental diffusion. The larger the molecular size and solubility of the lipid, the better is the placental transfer [67]. Substances delivered during the cleavage and blastula phases of mammalian embryonic development, as well as before implantation, which happens on the sixth day of gestation in rats, often elicit minimal teratogenic reaction, despite the fact that the same agents evoke noticeable responses when administered at higher dosages later in embryo development [68].

The embryo's vulnerability to teratogenesis decreases as tissue differentiation develops, and once organogenesis is complete, the embryo as a whole is teratogen-resistant [69]. As a result, TAZ administration in this investigation was limited to the critical period of organogenesis, which is the 6th–15th day of gestation, when cellular differentiation takes place and the rat embryo is most vulnerable to external and internal stimuli. The current study examined the effects of TAZ on growing embryo during pregnancy to the control group. It has been suggested that a drug's teratogenic effect can be predicted if it can bypass the placental barrier [70] or inhibit protein synthesis [71], as well as reduce the activity of the material enzymes [72].

Several factors may contribute to TAZ's effect on fetal growth and development. TAZ is metabolised by intestinal microorganisms into two metabolites: sulfanilic acid and aminopyrazolone [73]. These metabolites are destroyed slowly or not at all, and they can produce reactive oxygen species, which can cause abnormalities in the developing embryo [74]. Many xenobiotics cause oxidative stress, which contributes to their toxicity [75]. Furthermore, synthetic food colouring compounds, such as TAZ, have been shown to decrease mitochondrial respiration in rat liver and kidneys [76] and alter mitochondrial membrane integrity, which is critical for sustaining mitochondrial activities and causing cellular death. As a result, TAZ-induced embryonic deformities could be linked to an increase in apoptosis. This could be the reason for disruption of the mitochondria and inactivation of certain enzymes, which is concerned with the energy metabolism [77].

*(2) Adverse Effect*. [78]. Tartrazine is considered as a cheaper substitute for natural food colorants like curcumin and saffron and is the second most used food dye, generally derived from coal tar. Cardiomegaly, hepatorenal damage, and splenic pigmentation were also found in the TAZ-treated groups. In this view, dietary additive intake is strongly associated to mutagenicity in the form of gene mutation and chromosomal abnormalities [79]. In this study, the effects of tartrazine on developing embryo during the gestation period were compared to the control group. It has been proposed that a drug's teratogenic effect can be predicted if it can breach the placental barrier, diminish protein synthesis, and inhibit material enzyme function. Administration of toxicants produces multiorgan toxicity, even though it is organ specific [80].

The effect of tartrazine on fetal growth and development could be due to a number of variables [81]. In the fetuses, TAZ increased fetal resorptions and mortality, as well as cardiomegaly, hepatorenal damage, and splenic pigmentation. Missing coccygeal vertebrae, missing sternebrae, missing hind limbs, and unequal ribs were among the skeletal malformations caused by the treatment. TAZ was found to be embryotoxic and teratogenic in rats as a result of these findings [82].

### 3.5. Fortifying Agents as Teratogens

The practice of adding vitamins and minerals to regularly consumed foods during processing to increase their nutritional value is known as food fortification. It is a tried-and-true, safe, and affordable technique for improving diets and preventing and controlling micronutrient deficiencies. Cereals and cereal-based products, milk and dairy products, fats and oils, accessory food items, tea and other beverages, and newborn formulae are the most commonly fortified foods, according to the FAO. This procedure is used by food manufacturers to increase micronutrients and vitamins in their goods by adding food fortification agents. Food strengthening agents are utilized in staple foods to reduce dietary deficit. To boost the nutrients in dietary food and cereals, food-fortifying agents are used [83]. The increased demand for healthful foods is the primary driver of food-fortifying agents. Because of their changing lifestyles, consumers are becoming more conscious of healthy food products. There are numerous issues that function as roadblocks to the market expansion of food-fortifying agents.

#### 3.5.1. Vitamin A

Vitamin A is an essential component for pregnant mothers and their developing fetus [84]. Vitamin A fortification is thought to function by boosting daily intake and absorption of preformed vitamin A also called retinol (Figure 6) to levels adequate that close the current consumption gap and greatly increase liver reserves, hence correcting vitamin A deficiency and its health and survival implications is important. Since it is involved in cell differentiation, eye integrity maintenance, and the prevention of xerophthalmia, vitamin A plays a critical role in ocular function. Its absence is the leading cause of night blindness in the world. Vitamin A is necessary for the regular development of the embryo, in addition to its crucial role in numerous body tissues [85].

*(1) Mechanism of Action*. *In vitro* rat embryo studies have revealed that retinoids act directly on the embryo, causing abnormal development [86]. The quantity of active retinoid that accumulates over time (concentration-time relationship) during phases of organ development is important for developing organs. The rate at which retinoids are absorbed by the maternal intestine, maternal retinoid metabolism, the half-life of the retinoid in maternal plasma, and the rate at which retinoids are transferred from the pregnant female to her embryos are all factors that influence the amount of active retinoid in the embryo [87]. The effects of one retinoid may differ from one species to the next; each species has its unique animal tissue; thus, even when exposed to the same amount of retinoid, distinct developmental events may occur. By activating gene transcription in numerous areas of the embryo, retinoic acid aids in the regulation of embryonic development. The cells will only respond to retinoic acid if they have the appropriate receptors and retinoic acid concentrations are within the receptors' tolerable range. Many doctors and pathologists research the precise control of retinoic acid concentrations because varying levels of retinoic acid activate different genes. In the early phases of human embryonic development, notably the fourth week, retinoids help to promote the expression of Hox genes.

Hox genes are involved in the development of the embryo's body plan [88]. There are thirty-eight Hox genes in humans. The Hox gene malfunctions in embryos exposed to too much retinoic acid, disrupting the genetic control of body shape (axial patterning) during development [89]. Developmental abnormalities can result from these changes, notably in the embryonic spinal cord, central nervous system, and spinal cord, where retinoic acid production and catabolism enzymes are found. In 1953, Sidney Q. Cohlan discovered that high vitamin A doses in pregnant rats were linked to teratogens in the progeny.

*(2) Adverse Effects*. Vitamin A (retinol) is a vital vitamin for human health that aids in the regulation of epithelial tissue cellular development. Deformities in the fetuses' skulls, faces, limbs, eyes, and central nervous system can be observed in cases where pregnant women consume too much vitamin A and retinoid. Retinoids, which are vitamin A derivatives, are also extensively used to treat a range of skin problems, including carcinomas, which are the most common type of cancer in humans. Embryos from a range of animals, including monkeys, rabbits, rats, mice, and hamsters, were studied [90]. Central nervous system abnormalities such as an abnormally small head (microcephaly), incomplete development of the medulla spinalis (spina bifida), an encephalopathy in which some of the brain is found outside of the skull (exencephaly), and brain swelling due to fluid build-up were the most common defects found across all species (hydrocephaly). Facial nerve paralysis, underdevelopment of the upper jaw, cleft palate, cleft lip, nonexistent or malformed ears, and shortened limbs were among the other prevalent abnormalities, according to research [91].

## 4. Conclusion

The above-mentioned additives have teratogenic effect, so it must be replaced from our daily routine for better health. It can cause various health issues, so it is better to minimize the use of chemical food additives. In contrast to synthetic additives, natural food additives have gained wider acceptance due to their many advantages. According to the present study, chemical food additives can trigger a slew of serious health issues. The troubles that it creates will vary depending on the amount and duration of the preservatives used. Even if some additives do not act directly, they might nevertheless cause or contribute to health problems. The study also revealed how additives work, their mechanism of action, why they cause various health issues, and which health issues are caused by each synthetic food additives. Natural food additives help to extend the shelf life of a product while reducing the possibility of harmful side effects. Hence, natural food additives should be preferred over synthetic food additives.

## Figures and Tables

**Figure 1:** Chemical structure of sodium benzoate.

**Figure 2:** Chemical structure of potassium benzoate.

**Figure 3:** Chemical structure of aspartame.

**Figure 4:** Chemical structure of lambda carrageenan.

**Figure 5:** Chemical structure of tartrazine.

**Figure 6:** Chemical structure of retinol.

**Table 1:** Safety evaluation of certain food additives with examples and INS number.

S. no.	Functional class	Description	Example of food additive	INS no.	Acceptable daily intake (ADI)	Median lethal dose (LD_50_)
1.	Preservative	Prolong the shelf life of foods by protecting them against deterioration caused by microorganisms.	(a) Sodium benzoate (b) Potassium benzoate	211 212	0-5 mg/kg bw 0-5 mg/kg bw	Oral rat >4070 mg/kg [92] Rat >10,000 mg/kg [93]
2.	Sweeteners	Impart a sweet taste to foods or in tabletop sweeteners.	Aspartame	951	40 mg/kg bw	Oral rat >10,000 mg/kg [94]
3.	Stabilizers	Maintain the physicochemical state of a food stuff.	Carrageenan	407	75 mg/kg bw	Oral rat >5,000 mg/kg [95]
4.	Colouring agents	Add or restore colour in a food and include natural constituents of foods and natural sources.	Tartrazine	102	0-10 mg/kg bw	Mouse >6250 mg/kg [96]
